# Analysis of Clinical Characteristics and Risk Factors of Postoperative Recurrence and Malignant Transformation of Low-Grade Glioma

**DOI:** 10.1155/2022/4948943

**Published:** 2022-08-31

**Authors:** Cheng Luo, Qian Luo, Yaoduan Xu, Jiushan Song, Yi Liu, Laizang Wang, Zhuoqi Dong, Wei Huang, Hualin Yu, Jinghui Li

**Affiliations:** ^1^The Second Department of Neurosurgery, First Affiliated Hospital of Kunming Medical University, Kunming 650000, Yunan, China; ^2^The Department of Neurosurgery, Third People's Hospital of Honghe Prefecture, Gejiu 661000, Yunnan, China; ^3^The Pediatric Department, First Affiliated Hospital of Kunming Medical University, Kunming 650000, Yunnan, China

## Abstract

This research was developed to explore the clinical characteristics and related risk factors of postoperative recurrence and malignant transformation of low-grade glioma (LGG). The subjects were rolled into observation group (19 cases) and control group (51 cases) according to recurrence and malignant transformation during the follow-up period. The clinical data of the two groups were compared, and the risk factors of recurrence and malignant transformation were analyzed with the time of recurrence and malignant transformation as independent variables. The experimental results showed that the proportion of patients aged over 45 years in the observation group (63.16%) was higher than that in the control group (50.98%). The proportion of preoperative functional status score (KPS) ≥80 in the observation group (68.42%) was lower than that in the control group (78.43%). The proportion of patients with tumor over 5 cm in the control group (27.45%) was lower than that in the observation group (52.63%), and the proportion of total resection of tumor in the control group (47.06%) was higher than that in the observation group (21.05%). Furthermore, the multivariate analysis showed that preoperative KPS score, preoperative duration of disease, resection scope, postoperative treatment, oncotesticular antigen (OY-TES-1) mRNA, P53, mouse double microbody amplification gene (MDM2), vascular endothelial growth factor (VEGF), and epidermal growth factor receptor (EGFR) were independent risk factors (all *P* < 0.05). In summary, patients with postoperative recurrence and malignant transformation had poorer physical condition and higher degree of malignancy before surgery. Preoperative KPS score, duration of disease, surgical resection scope, postoperative treatment, OY-TES-1 mRNA, P53, MDM2, VEGF, and EGFR were the risk factors.

## 1. Introduction

Intracranial tumors are classified into primary and secondary types according to their specific causes. Tumor types are also different in different age groups. For younger children, intracranial tumors mainly occur in the posterior fossa and midline. For adults, it is mainly a glioma of the cerebral hemisphere [1]. The cerebral hemisphere is part of the brain that controls movement, language, and emotion. Gliomas occur in the cerebral hemisphere and can cause headaches, nausea, vomiting, seizures, and limb movement disorders. Glioma, as a primary intracranial tumor, has a high recurrence rate and fatality rate [2]. At present, the main clinical diagnosis methods are skull CT and nuclear magnetic examination. Existing studies suggested that glioma, as a malignant tumor, is mainly formed by intermutations between astrocytes, oligodendrocytes, ependymal cells, and neurons [3]. According to statistics, there are more male patients than female patients, and the age of patients is generally younger. The growth of mesenchymal tumors is usually slow, and the time from onset of symptoms to medical treatment is usually several weeks to several months and a few years. In addition, glioma has the possibility of metastasizing to other parts of the body [4], and the metastasis path generally occurs through the subarachnoid space, blood, and lymphatic system. The first is through the subarachnoid space. Medulloblastoma among gliomas is easily transplanted along the subarachnoid space and may induce tube meningiomas and intraorbital tumors. To avoid this kind of metastasis, it is necessary to have whole-brain or spinal cord radiation therapy after surgery. The second path of metastasizing the tumor is blood transfer. The most common way gliomas metastasize is through blood, through which patients can develop lung, breast, and skin cancers, and this route of metastasis is very difficult to prevent. The third way is metastasis through the lymphatic system. Glioma can also metastasize through the lymphatic system, and tumors may enter specific organs or parts of the body along the lymphatic space around spinal nerves or cranial nerves to induce diseases [5]. Because all parts of the body are lymphatic, this metastasis is very harmful to the body. To prevent lymphatic system metastasis, patients must actively take countermeasures after the occurrence of disease.

Gliomas include low-grade glioma (LGG) and high-grade glioma (HGG) according to their clinical characteristics and degree of malignancy [6]. LGG patients have slow disease progression and good postoperative prognosis. Although there is a possibility of recurrence, the overall chances of recurrence are less. HGGs develop rapidly, and relapse occurs in a short period of time after surgery [7]. Clinically, both intraoperative and postoperative images accurately showed that the tumor was removed, and then the tumor grew at the original site again, which was called recurrence [8]. However, recurrence is rare for LGG, and the main clinical findings are incomplete surgical resection and a small amount of residual tissue. Intraoperative neglect and postoperative image reflection are not obvious, with a small residual site, and continued growth leads to a second operation [9]. The tumor has an indistinct border with the surrounding brain tissue or is located in important functional areas. This tumor was conservatively excised for fear of damaging the surrounding functional areas. Some tumors are deep and have a poor surgical field of vision, resulting in residue. There are also large tumors that are left intraoperatively for different reasons, and these residues can also cause recurrence. Therefore, regular follow-up and even chemotherapy and radiotherapy are recommended to reduce the risk of recurrence. In addition, even though the postoperative prognosis of ground-based glioma is good, malignant transformation (MTF) also occurs in some patients [10]. MTF refers to LGG progression to World Health Organization (WHO) grade III or IV tumor [11]. According to the literature, the incidence of LGG MTF is 23–72%, and the median time of MTF is 2.7–5.4 years [12]. For patients with LGG, craniotomy under general anesthesia is often used for treatment. According to the patient's situation, maximum tumor resection or total tumor resection can be selected. However, due to the characteristics of diffuse growth, recurrence may occur after surgery, so postoperative radiotherapy and chemotherapy are generally used [13]. In addition, after surgical treatment, physical therapy, speech therapy, and other rehabilitation treatments can be carried out to avoid disease recurrence and prolong the survival time of patients. Since LGG can also be a high-grade glioma with MTF grade III or IV in the course of disease, regular dynamic follow-up observation is required even after surgery [14, 15].

Although LGG has a relatively good prognosis after surgery, there will be a certain possibility of recurrence and MTF if it is not prevented after surgery. If advanced glioma develops, it will pose a serious threat to the survival of patients. Therefore, understanding the postoperative recurrence of LGG and the clinical characteristics of MTF and grasping the related factors causing recurrence and MTF can prejudge the postoperative situation of patients to avoid the occurrence of such phenomena. In this experiment, the patients with LGG were followed up after surgery, the recurrence and MTF time of patients with recurrence and MTF were recorded, and the basic information of patients without progression of the disease was compared to obtain the clinical characteristics of patients with recurrence and MTF. The existing research data were reviewed to determine the relevant factors affecting the progression of the patient's disease and were included in the study scope to explore the risk factors related to relapse and MTF among the relevant factors. The above experiments are expected to provide a reference for the clinical prevention of postoperative recurrence and MTF in LGG patients.

## 2. Materials and Methods

### 2.1. Research Objects

Seventy patients who received LGG surgery in the Neurosurgery Department of the First Affiliated Hospital of Kunming Medical University from 2019 to 2021 were selected as the study subjects. There were 49 males and 21 females, ranging from 30 to 70 years old, with an average age of 42.7 ± 11.5 years. According to the diagnostic criteria of recurrence and malignant transformation, a total of 19 patients showed recurrence and malignant transformation, and the rate of recurrence and malignant transformation was 27.14%. According to the progress of postoperative disease, patients without postoperative disease changes were set as the control group, and patients with postoperative recurrence and malignant transformation were set as the observation group. This study had been approved by the Medical Ethics Committee of the First Affiliated Hospital of Kunming Medical University. Patients and their families understood the research content and methods and agreed to sign corresponding informed consent forms.

Inclusion criteria were as follows: (i) pathological diagnosis of LGG; (ii) patients aged ≥18 years; (iii) patients with complete clinical data.

Exclusion criteria were as follows: (i) patients with other tumors; (ii) patients with liver and kidney dysfunction; (iii) patients unwilling to cooperate with the whole follow-up process.

### 2.2. Research Methods

General information (sex, age, and preoperative physical status score), preoperative epilepsy and preoperative duration, tumor status (tumor size and tumor location), and related surgical treatment information (resection scope) of 70 patients who met the criteria were collected before surgery. Related protein levels after the operation, including proliferating cell nuclear antigen (PCNA), matrix metalloproteinase 9 (MMP-9), cancer testicular antigen OY-TES-1 protein, OY-TES-mRNA protein expression, P53, mouse double microsomal amplified gene MDM2, vascular endothelial growth factor (VEGF), and epidermal growth factor receptor (EGFR), were detected. Methods of treatment (chemotherapy, radiotherapy, and radiotherapy + chemotherapy), postoperative Karnofsky Performance Scale (KPS) score, epilepsy, and other conditions were analyzed. After that, patients were followed up. During the follow-up, patients' postoperative recovery was known by phone or text message, and the recurrence time of patients with recurrence and MTF was counted. Based on the above information, the clinical characteristics of patients with recurrence and MTF were analyzed, and the risk factors for recurrence and MTF were analyzed with the time of recurrence and MTF as independent variables. The related technical route or data collection of the research participants and concluding reports is shown in Figure 1.

### 2.3. Relative Protein Detection

The immunohistochemical streptomycin biotin-peroxidase method (SP) and polymerase chain reaction (PCR) were used to determine the expression of related proteins (Figure 2).

### 2.4. Observation Indicators

General data of the patients, including sex, age, preoperative KPS score, preoperative duration of disease, postoperative KPS score, and postoperative epilepsy, were collected.

Tumor conditions, such as tumor size and tumor location, were recorded.

Surgical treatment information, such as surgical resection scope and postoperative treatment, was collected.

Protein levels, including PCNA, MMP-9, OY-TES-1, OY-TES-mRNA, P53, MDM2, VEGF, and EGFR, were detected.

### 2.5. Statistical Methods

SPSS 22.0 was used for statistical analysis of the study. Measurement data were indicated as the mean ± standard deviation. The *X*^2^ (Chi-square) test was used for comparisons between groups, the Kaplan–Meier method was used for univariate analysis, and Cox regression analysis was used for multivariate analysis. *P* < 0.05 was considered statistically significant.

## 3. Results

### 3.1. General Information

The comparison of general data between the observation group and the control group showed that there were statistically significant differences in age, preoperative KPS score, and preoperative epilepsy between the two groups, *P* < 0.05. The proportion of patients aged over 45 years in the observation group was 63.16%, and that in the control group was 50.98%. The proportion of patients aged over 45 years in the observation group was higher than that in the control group. Of those with a preoperative KPS score ≥80, the observation group accounted for 68.42%, the control group accounted for 78.43%, and that of the observation group was less than that of the control group. The proportion of patients with epilepsy before surgery was 15.79% in the observation group and 35.29% in the control group, which was smaller in the observation group than that in the control group. The details are shown in Table 1.

### 3.2. Tumor Size and Location

The tumor size difference between the observation group and the control group was statistically significant, *P* < 0.05. The proportion of patients with tumor over 5 cm was 27.45% in the control group and 52.63% in the observation group, which was larger in the observation group than that in the control group. The details are shown in Table 2.

### 3.3. Comparison of Surgical Resection Range and Postoperative Treatment

The surgical resection range and postoperative treatment were compared between the two groups, and the differences were remarkable, *P* < 0.05. Total resection accounted for 47.06% in the Ctrl group and 21.05% in the Obs group, which was smaller in the Obs group than that in the Ctrl group. The proportion of patients receiving radiotherapy plus chemotherapy after surgery in the Ctrl group was 41.18%, and that in the Obs group was 15.79%, which was smaller in the Obs group than that in the Ctrl group (Table 3).

### 3.4. Relative Protein Expression

The positive expression of each protein was compared between the observation group and the control group, and the difference was statistically significant (all *P* < 0.05). The proportion of patients with positive PCNA expression was 37.25% in the control group and 94.74% in the observation group, which was smaller in the control group than that in the observation group. The proportion of MMP-9 positive patients was 15.69% in the control group and 100% in the observation group, which was smaller in the control group than that in the observation group. The proportion of patients with positive OY-TES-1 expression was 29.41% in the control group and 42.11% in the observation group, which was smaller in the control group than that in the observation group. The proportion of patients with positive OY-TES-mRNA expression was 33.33% in the control group and 47.37% in the observation group, which was smaller in the control group than that in the observation group. The proportion of patients with positive P53 expression was 49.02% in the control group and 89.47% in the observation group, which was smaller in the control group than that in the observation group. The proportion of MDM2 positive patients was 52.94% in the control group and 78.95% in the observation group, which was smaller in the control group than that in the observation group. The proportion of patients with positive VEGF expression was 33.33% in the control group and 57.89% in the observation group, which was smaller in the control group than that in the observation group. The proportion of patients with positive EGFR expression was 60.78% in the control group and 89.47% in the observation group, which was smaller in the control group than that in the observation group. The details are shown in Table 4 and Figure 3.

### 3.5. Risk Factor Analysis

Univariate analysis showed that preoperative KPS score, preoperative duration of disease, surgical resection scope, postoperative treatment, and expression of PCNA, OY-TES-1, OY-TES-mRNA, P53, MDM2, VEGF, and EGFR proteins were all related to recurrence and MTF in Obs group, all *P* < 0.05. Sex, age, tumor site, tumor size, postoperative KPS score, and postoperative epilepsy were not associated with recurrence or MTF (*P* > 0.05). The details of single factor analysis in the observation group are shown in Table 5. Cox regression analysis of *P* < 0.05 in univariate analysis showed that preoperative KPS score, preoperative duration of disease, surgical resection scope, postoperative treatment, and expression of OY-TES-mRNA, P53, MDM2, VEGF, and EGFR proteins were independent risk factors affecting recurrence and MTF, all *P* < 0.05. The details of the multifactor analysis of relapse and malignant transformation are shown in Table 6.

## 4. Discussion

Glioma is a tumor disease in neurosurgery. The most common clinical manifestation is tumor growth to a certain extent. It can cause obvious symptoms of high cranial pressure, which mainly manifest as headache, vomiting, and blurred vision. Other manifestations and secondary glioma growth areas have very large relations. If glioma grows in the motor area, it can cause contralateral limb activity obstacles. If glioma grows in the optic nerve, it can cause vision problems, tending to develop glioma in the cortex. If it involves the cortex, it can cause epilepsy [16]. The survival time of a patient with glioma mainly depends on the treatment, degree of malignancy of the tumor, and patient constitution. LGG refers to malignant LGG of the brain [17]. Generally, astrocytoma and oligodendroglioma have a good prognosis for LGG [18]. For LGG patients, craniotomy under general anesthesia is often used for treatment, and maximum tumor resection or total tumor resection is selected according to the patient's situation. Due to its characteristics of diffuse growth, there is a possibility of recurrence and MTF after surgery, so postoperative radiotherapy and chemotherapy are generally used [16]. In addition, after surgical treatment, physical therapy, speech therapy, and other rehabilitation treatments can be carried out to avoid disease recurrence and prolong the survival time of patients. LGG usually includes grade I gliomas and grade II gliomas. Grade I gliomas have low proliferative potential, are relatively confined, and can be cured by surgical resection. Grade II gliomas generally refer to invasive growth, which is characterized by low proliferative activity and a low degree of malignancy. However, if the degree of resection is insufficient, residual lesions will relapse and even develop into high-grade lesions, thus affecting life [6, 19]. Generally, LGG is more commonly seen in well-differentiated diffuse astrocytoma, also known as low-grade diffuse astrocytoma. The onset age is 30–40 years, and there are more males than females. In addition, CT neuroimaging examination shows low-density lesions with unclear inner edges of the brain, obvious enhancement, or cystic changes. MRI will display a relatively low signal in T1 and a relatively high space-occupying lesion in T2 [20]. Patients with LGG receive comprehensive treatment based on surgical resection, thus providing the possibility of long-term and high-quality survival. For some cases of relapse and MTF after treatment of glioma, this consideration is due to the following reasons. The first is environmental. If patients continue to go to places with high radiation levels after glioma treatment, the tumor cells will mutate again, and the disease will recede. The second is improper postcare. Care after glioma treatment is critical, and if the care is not appropriate, it is very easy to cause disease recurrence and malignant change. The third is that the operation excision is not clean. The postoperative progression of glioma may be caused by unclean surgical resection. The shape and location of glioma vary from person to person. The tumor location of some patients is special, and there may be many tissues or blood vessels around it. In this case, it is difficult to remove the tumor, and only part of the tumor may be removed, but not completely. This kind of glioma that is not completely resected needs adjuvant therapy after surgery to control tumor regrowth [21, 22]. If there is no postoperative adjuvant therapy, then the probability of glioma recurrence and MTF is very large. People who are susceptible to this disease in daily life are mainly the following: (i) people who have been infected with cytomegalovirus are more likely to suffer from this disease, but there is no conclusion at present; (ii) people with familial genetic factors are more prone to this disease; and (iii) people with long-term exposure to ionizing radiation are more likely to experience glioma. For example, they often use mobile phones and computers for a long time [23].

LGG patients can live up to 30 years if treated promptly. However, according to the current overall treatment results, it is still difficult to cure. According to statistics, the 5-year and 10-year survival rates of LGG patients are 60% and 35%, respectively, while the median survival period of LGG is between 8 and 10 years [24]. Therefore, understanding the clinical characteristics of postoperative recurrence and malignant transformation of LGG and grasping the related factors causing recurrence and malignant transformation can prejudge the postoperative situation of patients so as to avoid the occurrence of disease progression and reduce the survival time of patients. In this experiment, LGG patients were followed up after surgery, and the time of recurrence and malignant transformation of patients with recurrence and malignant transformation was recorded. Moreover, the basic information of patients without progression of disease was compared so as to obtain the clinical characteristics of patients with recurrence and malignant transformation. By referring to existing research data, the relevant factors affecting the progression of patients' disease were determined and included in the research scope, and the risk factors related to relapse and malignant transformation among the relevant factors were explored. The experimental results showed that the proportion of patients aged over 45 years in the observation group was 63.16%, and that in the control group was 50.98%. The proportion of patients aged over 45 years in the observation group was larger than that in the control group. It indicates that older patients are vulnerable to disease recurrence and malignant transformation due to the decline of autoimmune function and metabolic ability after surgery. KPS score is also known as the tumor patient quality of life score. Patients with a score greater than 80 performed well in all physical indicators [25]. In this experiment, the proportion of patients with preoperative KPS score ≥80 in the observation group was 68.42%, and that in the control group was 78.43%, which was smaller in the control group than that in the observation group. It indicates that patients with malignant progression of postoperative disease are mostly patients with poor physical condition before surgery. The proportion of patients with epilepsy before surgery was 15.79% in the observation group and 35.29% in the control group, which was smaller in the observation group than that in the control group. It was found that the mechanism of epilepsy induced by glioma may be that the invasive tumor cells change the excitability of the surrounding normal neurons, making them the pacemakers of seizures. However, the destructive effect of malignant tumors on peripheral neurons and their axons obstructs the occurrence and transmission of epilepsy [26, 27]. In addition, patients with tumor over 5 cm accounted for 27.45% in the control group and 52.63% in the observation group, which was larger in the observation group than that in the control group. The malignant degree of disease was higher in patients with disease progression after operation. The total resection accounted for 47.06% in the control group and 21.05% in the observation group, which was smaller in the observation group than that in the control group. Meanwhile, the postoperative radiotherapy plus chemotherapy accounted for 41.18% in the control group and 15.79% in the observation group, which was smaller in the observation group than that in the control group. These results indicate that the patients with disease progression after surgery were mostly patients with incomplete surgical resection and single postoperative adjuvant therapy. Tumor markers can indicate the existence and growth of tumors, and monitoring tumor markers can help judge the treatment effect, prognosis, recurrence, and metastasis [28]. Proliferating cell nuclear antigen (PCNA) was first identified and named by Miyachi in 1978 in sera from patients with systemic lupus erythematosus (SLE). In the scholar's study, PCNA was found to be closely related to cell DNA synthesis and played an important role in the initiation of cell proliferation, which was a good indicator of cell proliferation status. Therefore, PCNA research has been very hot in recent years, especially in the field of cancer. In this experiment, the proportion of patients with positive PCNA expression was 37.25% in the control group and 94.74% in the observation group, which was smaller in the control group than that in the observation group. MMP-9 is an enzyme belonging to the zinc-metalloproteinase family. In this study, the proportion of MMP-9 positive patients was 15.69% in the control group and 100% in the observation group, which was smaller in the control group than that in the observation group. As a tumor marker, the expression of cancer testicular antigen OY-TES-1 mRNA was generally low in normal tissues and high in cancer lesion tissues. In this study, the proportion of patients with positive OY-TES-mRNA expression was 33.33% in the control group and 47.37% in the observation group, which was smaller in the control group than that in the observation group. Since its discovery in 1979, P53 has been a focus of oncology research. P53 is a tumor suppressor gene, and P53 mutations occur in many tumors, so it is common to see reports of immunohistochemical staining of P53 in tumors. In this study, the proportion of patients with positive P53 expression was 49.02% in the control group and 89.47% in the observation group, which was smaller in the control group than that in the observation group. MDM2 has been found to be amplified and expressed in a variety of tumors and can coadjust with P53 tumor suppressor gene to promote tumor formation and development. In this study, the proportion of MDM2-positive patients was 52.94% in the control group and 78.95% in the observation group, which was smaller in the control group than that in the observation group. EGFR, which plays an important role in physiological processes such as cell growth, proliferation, and differentiation, is overexpressed in a variety of solid tumors. VEGF plays an important role in angiogenesis, invasion, and metastasis of various tumors. In this study, the proportion of patients with positive VEGF expression was 33.33% in the control group and 57.89% in the observation group, which was smaller in the control group than that in the observation group. The proportion of patients with positive EGFR expression was 60.78% in the control group and 89.47% in the observation group, which was smaller in the control group than that in the observation group. The above protein expression results indicate that patients with postoperative recurrence and malignant transformation also have a higher positive rate of related tumor markers. Furthermore, the single factor analysis of the related factors causing the progression of postoperative disease showed that preoperative KPS score, preoperative duration of disease, surgical resection scope, postoperative treatment, and PCNA, OY-TES-1, OY-TES-mRNA, P53, MDM2, VEGF, and EGFR protein expression were all related to recurrence and malignant transformation (all *P* < 0.05). Multivariate analysis showed that preoperative KPS score, preoperative duration of disease, surgical resection scope, postoperative treatment, and expression of OY-TES-mRNA, P53, MDM2, VEGF, and EGFR proteins were independent risk factors affecting recurrence and malignant transformation (all *P* < 0.05).

## 5. Conclusion

The clinical characteristics of postoperative recurrence and MTF in LGG patients were older patients, lower preoperative KPS score, larger tumor, incomplete surgical resection, single postoperative treatment, and higher preoperative malignancy. Independent risk factors included preoperative KPS score, preoperative duration of disease, surgical resection scope, postoperative treatment, and expression of OY-TES-mRNA, P53, MDM2, VEGF, and EGFR proteins.

## Figures and Tables

**Figure 1:** Technical route for data collection of the research participants and concluding reports.

**Figure 2:** Related protein expression detection process through PCR and SP immunohistochemistry methods.

**Figure 3:** Expression of related proteins in primary, recurrent, and malignant transformed gliomas (SP400×). Note: a1, a2, b1, b2, c1, c2, e1, e2, f1, f2, g1, g2, and h1, h2 are the levels of PCNA, MMP-9, OY-TES-1, P53, MDM2, VEGF, and EGFR in primary and malignant transforming gliomas, respectively. d is the positive expression of OY-TES-1 mRNA, where 1 is DNA marker, 2 is testicular cDNA (positive control), 3 is positive expression of OY-TES-1 mRNA in primary glioma tissues, and 4–6 are positive expression of OY-TES-1 mRNA in recurrent and MTF glioma tissues.

**Table 1:** Comparison of general data between the two groups.

Information	Ctrl group (*n* = 51)	Obs group (*n* = 19)	X^2^	*P*
Sex			0.098	0.867
Male	35	14		
Female	16	5		

Age			5.465	0.026
≤45	25	7		
>45	26	12		

Preoperative KPS score			7.836	0.013
<80	11	6		
≥80	40	13		

Preoperative epilepsy			4	0.024
Yes	18	3		
No	33	16		

Preoperative duration of disease (month)			0.113	0.076
≤3	14	5		
3–6	27	7		
>6	10	7		

**Table 2:** Comparison of tumor-related conditions between the two groups.

Type	Group		*X* ^2^	*P*
	Ctrl group	Obs group		
*Tumor site*				
Cerebral hemisphere	38	13	0.223	0.572
Others	13	6		

*Tumor size (cm)*				
≤5	37	9	5.184	0.037
>5	14	10		

**Table 3:** Surgical resection range and postoperative treatment comparison between the two groups.

Type	Group		*X* ^2^	*P*
	Ctrl group	Obs group		
*Surgical resection range*				
Total resection	24	4	6.962	0.021
Subtotal resection	15	7		
Local total resection	12	8		

*Postoperative treatment*				
Radiation therapy	14	9	5.134	0.028
Chemotherapy	16	7		
Radiotherapy + chemotherapy	21	3		

**Table 4:** Positive comparison of related protein expression between the two groups.

Type	Group		*X* ^2^	*P*
	Ctrl group (*n* = 51)	Obs group (*n* = 19)		
PCNA	19 (37.25%)	18 (94.74%)	4.596	0.035
MMP-9	8 (15.69%)	19 (100%)	6.812	0.005
OY-TES-1	15 (29.41%)	8 (42.11%)	3.563	0.041
OY-TES-1 mRNA	17 (33.33%)	9 (47.37%)	5.977	0.022
P53	25 (49.02%)	17 (89.47%)	9.856	0.001
MDM2	27 (52.94%)	15 (78.95%)	7.263	0.030
VEGF	17 (33.33%)	11 (57.89%)	5.160	0.017
EGFR	31 (60.78%)	17 (89.47%)	4.035	0.039

**Table 5:** Single factor analysis of recurrence and malignant transformation in the Obs group.

Type	Cases of recurrence and malignant transformation	Mean time to recurrence and malignant transformation (months)	*t*	*P*
*Sex*				
Male	14	21.69 ± 2.13	−0.081c	0.987
Female	5	23.56 ± 1.58		

*Age*				
≤45	7	24.23 ± 2.54	−0.795	0.524
>45	12	21.77 ± 2.36		

*Preoperative KPS score*				
<80	6	15.02 ± 2.13	4.846	0.046
≥80	13	22.67 ± 2.61		

*Preoperative duration of disease (month)*				
≤3	5	15.13 ± 1.54	4.563	0.003
3–6	7	13.61 ± 2.99		
>6	7	9.75 ± 3.32		

*Tumor site*				
Half of the brain	13	19.86 ± 2.31	0.522	0.087
Others	6	14.12 ± 2.04		

Tumor size (cm)				
≤5	9	23.75 ± 3.46	0.565	0.325
>5	10	20.91 ± 2.78		

*Surgical resection range*				
Total resection	4	20.05 ± 2.06	11.042	0.036
Subtotal resection	7	18.47 ± 2.35		
Local total resection	8	13.32 ± 2.89		

*Postoperative KPS score*				
<80	8	10.02 ± 2.54	0.786	0.261
≥80	11	12.58 ± 2.96		

*Preoperative epilepsy*				
Yes	3	12.35 ± 1.86	0.092	0.872
No	16	10.78 ± 2.05		

*Postoperative treatment*				
Radiation therapy	9	9.56 ± 2.16	3.746	0.023
Chemotherapy	7	10.48 ± 1.88		
Radiotherapy + chemotherapy	3	13.59 ± 2.04		

*PCNA expression*				
Negative	1	14.12 ± 2.84	3.976	0.031
Positive	11	11.04 ± 3.10		
Strong positive	7	8.67 ± 2.55		

*MMP-9 expression*				
Positive	8	12.83 ± 3.56	0.495	0.043
Strong positive	11	9.86 ± 3.28		

*OY-TES-1 protein expression*				
Negative	11	20.62 ± 2.43	3.562	<0.001
Positive	8	27.54 ± 2.61		

*OY-TES-1 mRNA protein expression*				
Negative	10	19.85 ± 2.79	3.336	<0.001
Positive	9	26.93 ± 3.15		

*P53*				
Negative	2	23.41 ± 2.09	2.875	0.003
Positive	17	11.26 ± 2.54		

*MDM2*				
Negative	4	22.43 ± 3.24	3.594	0.026
Positive	15	16.68 ± 3.38		

VEGF				
Negative	8	19.64 ± 3.08	3.119	0.009
Positive	11	15.44 ± 2.61		

*EGFR*				
Negative	2	20.15 ± 2.87	2.967	0.043
Positive	17	13.47 ± 2.64		

**Table 6:** Multifactor analysis of relapse and malignant transformation.

Item	Parameter estimates	The standard deviation	Wald *X*^2^	*P*
Preoperative KPS score	0.650	0.361	6.489	0.032
Preoperative duration of disease	1.269	0.359	5.419	0.027
Surgical resection range	0.631	0.204	9.206	0.003
Postoperative treatment	0.725	0.435	4.086	0.041
PCNA	1.123	0.608	3.564	0.065
OY-TES-1	1.232	0.713	3.385	0.078
OY-TES-1 mRNA	0.657	0.579	4.513	0.034
P53	0.656	0.198	7.897	0.006
MDM2	0.631	0.294	6.261	0.003
VEGF	1.104	0.328	4.266	0.020
EGFR	0.827	0.211	9.581	0.004

## Data Availability

The data used to support the findings of the study can be obtained from the corresponding author upon request.
